# The Efficacy and Safety of Plasma Exchange in the Treatment of Thrombotic Thrombocytopenic Purpura

This article has been retracted.

**DOI:** 10.1155/2022/3519937

**Published:** 2022-03-31

**Authors:** Zhilan Pan, Zhimin Zhang, Yan Yang, Weihua Hao

**Affiliations:** ^1^Blood of Internal Medicine, Shijiazhuang People's Hospital, Shijiazhuang 050000, Hebei Province, China; ^2^Cardiac Intensive Care Ward (CCU), Shijiazhuang People's Hospital, Shijiazhuang 050000, Hebei Province, China

## Abstract

**Background:**

Thrombotic thrombocytopenic purpura (TTP) is a clinically rare thrombotic cardiovascular and microvascular disease. The purpose of this study was to observe the clinical efficacy and safety of plasma exchange in the treatment of TTP.

**Methods:**

A total of 16 TTP patients who underwent plasma exchange from January 2015 to December 2020 were selected. The clinical data of all patients were collected for retrospective analysis. The effective rate of treatment, the changes of blood cell count before and after treatment, and adverse reactions during treatment were analyzed.

**Results:**

A total of 50 plasma exchanges were performed in 16 TTP patients. After plasma exchange treatment, there were 4 invalid and 12 improved patients. The total effective rate of plasma exchange in patients with TTP was 75.0%. After treatment, platelet count (PLT) and hemoglobin (Hb) levels were significantly increased in TTP patients. Compared with before treatment, lactate dehydrogenase (LDH), indirect bilirubin (IBIL), total bilirubin (TBIL), and broken red blood cells were significantly reduced. In addition, 3 adverse reactions occurred in 50 plasmapheresis procedures, and the incidence of adverse reactions was 6.0%.

**Conclusion:**

Plasma exchange therapy has a good therapeutic effect on TTP and can significantly improve abnormal blood cell count in patients with high safety.

## 1. Introduction

Thrombotic thrombocytopenic purpura (TTP) is a thrombotic microvascular disease characterized by the widespread formation of platelet thrombi in the microvessels. The disease has rapid onset, rapid progression, and high mortality [1]. TTP is a diffuse thrombotic microangiopathy. The disease is more common clinically, with a typical triad of thrombocytopenia, microangiopathic hemolytic anemia, and neuropsychiatric symptoms. If it is accompanied by fever and renal dysfunction, it is the classic pentad of TTP [2]. In the past, TTP had a poor prognosis and a short course of disease. To make matters worse, the mortality rate is 80% to 90% [3].

The etiology and pathogenesis of TTP have not been fully elucidated. Current studies have shown that the pathogenesis of TTP is related to the reduction or loss of ADAMTSl3 activity [4]. When ADAMTSl3 activity is decreased or lost, the excessive ultra-large von Willebrand factor polymer (UL-VWFM) secreted by vascular endothelial cells cannot be dissolved and cleared, resulting in the emergence of TTP [5]. The first onset of TTP is mainly in adults, with a male-to-female ratio of 1 : 2 [6]. According to the etiology, it can be divided into hereditary TTP and acquired TTP. The underlying disease of hereditary TTP is a mutation in the ADAMTS13 gene [7]. According to the etiology, acquired TTP can be divided into primary and secondary TTP. Primary TTP generally has no obvious cause, while secondary TTP is often secondary to autoimmune diseases, pregnancy, organ transplantation, drugs, infections, tumors, and other diseases [8].

In recent years, plasma exchange has been widely used in clinical practice, which can effectively reduce the mortality of TTP patients [9]. The principle of plasmapheresis is to separate and filter out the patient's plasma components through extracorporeal circulation and discard the patient's abnormal plasma components, thereby removing pathogenic substances, metabolites, and toxins in the patient's plasma. The typing components of the blood, supplemented albumin, and plasmapheresis fluid are then injected back into the patient [10,11]. Plasmapheresis can remove pathogenic factors in blood circulation and improve immune function [12]. During plasmapheresis, patients may experience adverse reactions such as plasma hypersensitivity, hypotension, and hypocalcemia [13].

This study selected 16 patients diagnosed with TTP from January 2015 to December 2020 as the research subjects. This study aimed to investigate the clinical efficacy and safety of plasma exchange in the treatment of TTP.

## 2. Materials and Methods

### 2.1. Patients

A total of 16 patients with TTP in Shijiazhuang People's Hospital from January 2015 to December 2020 were selected. The diagnostic criteria of TTP are based on the Chinese Expert Consensus on the Diagnosis and Treatment of Thrombotic Thrombocytopenic Purpura (2012 Edition). Among the 16 TTP patients, 6 were male (37.5%, 6/16) and 10 were female (62.5%, 10/16). Patients ranged in age from 23 to 64 years, with a median age of 44. Of the 16 TTP patients, 6 had systemic lupus erythematosus (SLE) and 2 had connective tissue disease. The triad of thrombocytopenia, microangiopathic hemolytic anemia, and neurological symptoms occurred in 11 patients (68.75%, 11/16). Five patients (31.25%, 5/16) developed a typical pentad of fever, renal impairment, thrombocytopenia, microangiopathic hemolytic anemia, and neurological symptoms. The general characteristics of the patients are shown in Table 1. This study was approved by the Medical Ethics Committee of Shijiazhuang People's Hospital.

### 2.2. Plasma Exchange Therapy

Plasma exchange therapy is used to treat patients diagnosed with TTP. Disposable plasmapheresis separation lines (Terumo BCT, USA) were routinely installed and prefilled with normal saline. Plasma exchange treatment parameters were set on a COBESpectra cell separator (Terumo BCT, USA) according to the patient's height, weight, and hematocrit. Generally, the replacement plasma volume is set at (40–50) mL/kg. A plasma exchange procedure was performed using albumin (15–25 g albumin in 500 mL of normal saline) and fresh frozen plasma as the replacement fluid. ACD-A (Sichuan Nangel) was used as anticoagulant, and the ratio of whole blood to anticoagulant was adjusted to 12–14. To prevent hypocalcemia during plasma exchange, 1–2 g of calcium gluconate is routinely supplemented during exchange. The changes of patient's vital signs were monitored during plasmapheresis, and the adverse reactions were conducted in a timely manner.

### 2.3. Other Treatments

In addition to plasma exchange, all 16 TTP patients received glucocorticoids. Six patients with TTP and SLE were treated with glucocorticoids, cyclophosphamide, and gamma globulin to control primary disease SLE. According to the specific clinical situation of each TTP patient, symptomatic and supportive treatment, such as transfusion of suspended red blood cells, anti-infection, acid suppression, hemostasis, and fluid replacement, were taken.

### 2.4. Efficacy Evaluation

Based on the “Diagnosis and Efficacy Criteria for Hematological Diseases,” the clinical efficacy of TTP patients was evaluated according to the improvement of platelet level and clinical symptoms after treatment.

Complete remission: after treatment, PLT≥150 × 10^9^/L, and clinical symptoms were significantly improved.

Improvement: PLT≥50 × 10^9^/L～＜150 × 10^9^/L, the increase of PLT is more than 100%, and the clinical symptoms are not improved obviously.

Invalid: after treatment, PLT <50 × 10^9^/L, the increase of PLT is less than 100%, and the clinical symptoms worsen.

The total effective rate = (the total number of cases−the number of invalid cases)/the total number of cases × 100%.

### 2.5. Observation Indicator

Hemoglobin (Hb), platelet count (PLT), broken red blood cell ratio, indirect bilirubin (IBIL), total bilirubin (TBIL), blood urea nitrogen (BUN), creatinine (Cr), and lactate dehydrogenase (LDH) levels were recorded before and after plasma exchange. The occurrence and treatment of adverse reactions during plasma exchange were recorded.

### 2.6. Statistical Analysis

Statistical analysis was performed using the statistical software SPSS17.0. All experiments were performed in 3 replicates. Before and after plasma exchange, Hb, the proportion of broken red blood cells, and LDH were analyzed using paired *t*-test. Data were expressed as mean ± SD. PLT, IBIL, TBIL, BUN, and Cr before and after plasma exchange were expressed as median *M* (P25–P75), and Wilcoxon signed rank test was used. *p* < 0.05 was considered statistically significant.

## 3. Results

### 3.1. The Frequency and Effective Rate of Plasma Exchange in TTP Patients

As shown in Figure 1, 7 patients underwent 3 plasmapheresis procedures. Five patients underwent two rounds of plasmapheresis. Two patients received one plasmapheresis. One patient received 7 cycles of plasma exchange. One patient underwent 10 cycles of plasmapheresis. Among the 16 TTP patients, 4 were ineffective and 12 were improved. The total effective rate of plasma exchange in 16 TTP patients was 75% (Table 2).

### 3.2. Blood Volume of Single Plasma Exchange in TTP Patients

As shown in Figure 2, the mean values of total circulating blood volume, exchanged plasma volume, fresh frozen plasma volume, and anticoagulant in a single plasma exchange in the 16 TTP patients were 4502 ± 563, 2318 ± 302, 2015 ± 236, and 397 ± 48 mL, respectively.

### 3.3. Comparison of Blood and Biochemical Parameters before and after Plasmapheresis

Next, blood and biochemical parameters were compared before and after plasmapheresis. We found that PLT and Hb were significantly increased after plasmapheresis compared with before treatment (*p* < 0.05, Table 3). Meanwhile, LDH, IBIL, TBIL, and broken red blood cells were significantly reduced after plasmapheresis compared with before treatment (*p* < 0.05, Table 3). Although Cr and BUN were also decreased after plasmapheresis, the differences were not significant compared with those before treatment (*p* ＞ 0.05, Table 3).

### 3.4. Adverse Reactions during Plasmapheresis

In this study, 16 TTP patients underwent a total of 50 plasmapheresis procedures. One patient developed chest tightness and palpitations during plasma exchange, and blood pressure dropped to 72/44 mmHg. After emergency intravenous infusion of 500 mL of hydroxyethyl starch and sodium chloride injection, 500 mL of 0.9% sodium chloride injection, 600 mL of plasma, and 20 mg of dopamine, the patient's blood pressure returned to normal and the symptoms disappeared. Another patient developed palpitations during 1 plasma exchange, and blood pressure dropped to 84/54 mmHg. After reducing the plasma exchange flow rate to 20 mL/min and infusion of 200 mL of plasma, the patient's blood pressure returned to normal and the symptoms disappeared. Another patient developed pruritus and erythema on the face and neck during 1 plasma exchange. After intramuscular injection of promethazine injection 12.5 mg and intravenous infusion of dexamethasone 5 mg, the patient's symptoms were relieved and plasma exchange was successfully completed. A total of 3 adverse reactions occurred in 50 plasma exchanges, and the incidence of adverse reactions was 6.0%.

## 4. Discussion

TTP is a rare blood disorder with an annual incidence of about one in a million. TTP can be divided into hereditary TTP and acquired TTP. Acquired TTP is further divided into primary TTP and secondary TTP [14]. Among the 16 patients in this study, 9 had primary TTP (56.25%, 9/16) and 7 had secondary TTP (43.75%, 7/16). Among them, 6 cases were secondary to SLE, accounting for 85.71% of secondary TTP. SLE is an autoimmune disease formed by antibodies and immune complexes that mediate organ tissue damage [15]. SLE is more common in women, accounting for 90% [16]. The male-to-female ratio of TTP patients in this study was 3 : 5, indicating that TTP is also more common in females. These results suggest that clinicians should be alert to the possibility of secondary TTP when treating SLE.

Typical clinical symptoms in TTP patients are the triad of thrombocytopenia, microangiopathic hemolytic anemia, and neurological symptoms [17]. In this study, the classic triad was present in 68.75% of the patients, and the pentad was present in 31.25% of the TTP patients. It is worth noting that some SLE patients have symptoms similar to TTP, which undoubtedly increases the difficulty of clinical diagnosis of TTP [18]. Therefore, these patients will be at risk of being missed or misdiagnosed. Some researchers believe that increased fragmented red blood cells (fragmented red blood cells ratio >1%), decreased Hb, decreased PLT count, and elevated serum LDH level are important basis for the diagnosis of TTP [19]. This study found that the PLT and Hb of the patients after plasma exchange were significantly increased, and the LDH and broken red blood cells of the patients were significantly decreased. The results show that plasma exchange has a good curative effect on TTP patients.

Due to the lack of effective treatment methods, the fatality rate of TTP patients is as high as 90% for a long period of time [20]. Around the 1960s, the mortality rate of TTP was decreased significantly when plasmapheresis was applied to the treatment of TTP. Plasma exchange is now recommended as first-line therapy for TTP [21]. Plasma exchange therapy should be initiated as soon as a patient is diagnosed or highly suspected of TTP [22]. In this study, 16 patients were treated with plasma exchange after a diagnosis of TTP. The number of plasma exchanges was 1 to 10 times, and the amount of plasma per exchange was (40–50) mL/kg. After plasma exchange, 12 patients recovered. The effective rate of plasma exchange for TTP was 75.0%. In this study, 16 patients with TTP underwent a total of 50 plasmapheresis procedures. Among them, adverse reactions occurred in patients during 3 plasma exchange procedures, and the incidence of adverse reactions was 6.0%. Among them, hypovolemic reactions accounted for 66.7%, and allergic reactions accounted for 33.3%. After corresponding clinical treatment, the patient's adverse reactions disappeared or alleviated. In view of the possible adverse reactions during plasma exchange, the treating physician needs to monitor the patient's physical condition during plasma exchange [23] to ensure the safety of the patients during treatment. However, the number of cases in this study is low. In the future, we still need to expand the number of cases to further verify our conclusions.

## 5. Conclusion

In conclusion, plasma exchange is effective means for the treatment of TTP. Once TTP is diagnosed or suspected, patients should be treated with plasma exchange as soon as possible. During treatment, doctors should monitor the occurrence of adverse reactions in TTP patients, deal with adverse reactions in a timely manner, and ensure the safety of patients during plasma exchange.

## Figures and Tables

**Figure 1:** List of plasma exchange times and corresponding cases in TTP patients. The number in figure means the number of cases (*n* = 16).

**Figure 2:** The mean data of single plasma exchange treatment in TTP patients (*n* = 16).

**Table 1:** General information of the patients.

Patients	Gender	Age	Weight	General symptoms and signs of the patient	Clinical diagnosis
1	Male	26	64	Fatigue, poor appetite, anemia, poor spirits	TTP
2	Female	63	48	Headache, fatigue, anemia, scattered bleeding spots all over the body	Connective tissue disease, TTP
3	Female	58	65	Fatigue and anorexia, sudden syncope 3 days ago, anemia, poor spirit	TTP
4	Male	64	56	Fever, chest tightness and fatigue, severe anemia	SLE, TTP
5	Female	24	60	Thrombocytopenia for more than 20 days, scattered petechiae and ecchymosis on the skin	TTP
6	Female	50	64	Fever, a little scattered purpura on the skin of the extremities, anemia	SLE, TTP
7	Male	51	70	Fever with thrombocytopenia for 1 week, scattered petechiae on both upper extremities, anemia	SLE, TTP
8	Female	35	55	Skin petechiae and ecchymosis, disturbance of consciousness for 1 day, irritability, anemia	TTP
9	Female	34	56	Thrombocytopenia, right upper quadrant tenderness, anemia	TTP
10	Female	45	47	Body petechiae and ecchymosis, convulsions with disturbance of consciousness for 1 day, anemia	SLE, TTP
11	Male	44	62	Petechiae and ecchymosis on both lower extremities, convulsions for 1 day, anemia	TTP
12	Female	30	45	Fever, thrombocytopenia, dizziness, fatigue, anemia	SLE, TTP
13	Female	56	68	Thrombocytopenia, abdominal discomfort, petechiae and ecchymosis, anemia	TTP
14	Male	23	44	Fever for 1 week, severe anemia, scattered petechiae and ecchymosis on the skin	SLE, TTP
15	Male	28	46	Left occipital paroxysmal pain with no apparent cause	TTP
16	Female	46	63	Increased menstrual flow, convulsions for 1 day, anemia	TTP

**Table 2:** The frequency and effective rate of plasma exchange in 16 TTP patients.

Patients	Number of plasma exchanges	Curative effect
1	1	Invalid
2	3	Improved
3	10	Improved
4	3	Invalid
5	1	Improved
6	2	Invalid
7	2	Improved
8	3	Improved
9	3	Improved
10	2	Improved
11	3	Improved
12	2	Improved
13	7	Invalid
14	2	Improved
15	3	Improved
16	3	Improved

**Table 3:** Comparison of blood and biochemical parameters before and after plasmapheresis.

Parameters	Before plasmapheresis	After plasmapheresis	*p* value
Hb (g/L)	62.95 ± 12.26	85.13 ± 19.21	*p* < 0.05^*∗*^
Broken red blood cells (%)	4.15 ± 1.84	2.01 ± 0.81	*p* < 0.05^*∗*^
LDH (U/L)	1024 ± 436	356 ± 174	*p* < 0.05^*∗*^
PLT (×10^9^/L)	9 (5–24)	115 (24–163)	*p* < 0.05^*∗*^
IBIL	40 (16.24–27.02)	7.23 (4.68–9.02)	*p* < 0.05^*∗*^
TBIL	34.52 (25.12–42.01)	13.47 (8.37–28.96)	*p* < 0.05^*∗*^
BUN (mmol/L)	8.15 (6.13–12.35)	5.26 (4.58–9.46)	*p* ＞ 0.05
Cr (*μ*mol/L)	73 (56–102.3)	55.64 (44.5–88.25)	*p* ＞ 0.05

## Data Availability

The data used to support the findings of this study are available from the corresponding author upon request.
